# Health View to Decrease Negative Effect of High Heels Wearing: A Systemic Review

**DOI:** 10.1155/2021/6618581

**Published:** 2021-03-12

**Authors:** Meizi Wang, Ci Jiang, Gusztáv Fekete, Ee-Chon Teo, Yaodong Gu

**Affiliations:** ^1^Faculty of Sports Science, Ningbo University, Ningbo, China; ^2^Faculty of Engineering, University of Pannonia, Veszprem, Hungary; ^3^Savaria Institute of Technology, Eötvös Loránd University, Hungary

## Abstract

Effective recommendations about how to decrease adverse effects of high heels (HH) need to be provided, since wearing HH is inevitable for most women in their daily life, regardless of their negative impacts on the foot morphology. The main purpose of this systematic review was to summarize studies which have provided specific information about how to effectively offset the negative effects of wearing HH, in the case of women, by means of examining heel height, insole, and heel base support (HBS). Some evidence indicate the following: (i) the range of appropriate heel height for HH shoes is 3.76 cm to 4.47 cm; (ii) compared to small HBS, the larger ones effectively increase gait stability, reduce risk of ankle injury, and improve comfort rating during HH walking; and (iii) the use of a total contact insert (TCI) significantly decreases plantar pressure and the impact on the foot, resulting in higher perceived comfort. It must be noted that these results are based on short-term research; therefore, any conclusions with regard to effects in the long term should be taken with a grain of salt. Nevertheless, future studies should be aimed at combining numerical and experimental methods, in order to provide personal recommendations for HH shoes by considering heel height and HBS size, based on the individual characters (weight, height, and age).

## 1. Introduction

The potential impact of HH shoes on women's health for over 50 years has been of concern in medical circles. Studies have shown that wearing HH can lead to slower self-selected walking speed, shorter step length, and smaller stance phase duration, while it increases ankle plantar flexion, knee plantar flexion, anterior pelvic tilt, and trunk extension [1–7]. Redistributing the plantar pressure, higher ground reaction forces (GRF), larger loading rate, higher peak knee external adduction moments, and higher peak patellofemoral joint stress have been detected during walking in HH [8–11]. It is worthy to note that substantial bodily adjustments have been observed due to wearing HH, e.g., change in the neuromuscular activation pattern, shortening of the gastrocnemius muscle fascicle muscles, increase in the Achilles tendon stiffness, and higher muscle activity of the soleus, tibialis anterior, and medial gastrocnemius [12–14]. These above-mentioned disturbances have been identified as negative implications for the human body. It is presumed that they contribute to several pathologies including metatarsalgia, hallux valgus, Achilles tendon tightness, knee osteoarthritis (OA), plantar fasciitis, and lower back pain, not to mention the elevated instability and imbalance, which can result in a greater risk of falling and slipping [15–19].

Despite widespread warnings from public health institutions and international medical societies [20], there is still a large proportion of the population wearing HH in their daily life. Regarding why women choose to wear HH, Broega et al. surveyed 574 females, between the ages of 24 and 45, who indicated that beauty and femininity were the key drivers of women's behavior [21]. Therefore, accurate suggestions must be provided about how to counter the adverse effects of HH using, instead of only giving a simple advice on not wearing it. Consequently, in the near future, the design of HH shoes must be associated to comfort and aesthetics in order to meet the requirements of beauty and health.

Up to now, researchers have made significant efforts to improve comfort of high-heeled shoes by suggesting a suitable heel height, an appropriate insert insole, sufficient support area of the heel, and even walking speed during HH gait. Studies have shown that an optimal range of height for maintaining postural balance and stability is between 3 and 5 cm [2, 17, 18]. Yung and Wei observed that a TCI, coupled with a metatarsal pad, arch support, and heel-cup mechanism, redistributed the plantar pressure, and as a consequence, it decreased the impact force by 33.2% in the case of HH [22]. It was also considered that small HBS increased the deviation of the center of pressure (COP), which on the one hand caused larger foot pressure in the rearfoot region, and on the other hand, it disturbed the muscle activity pattern [22].

However, the effects of physiology and ergonomics on HH design in terms of heel height, contact insole, and HBS have not yet been summarized. It is essentially needed to reach a consensus for shoe manufacturers and users on what kind of high-heeled shoes or insole is most optimal for women. Therefore, this systematic review is aimed at concluding studies that have provided a specific way to effectively offset the negative effects of wearing HH in the case of women. Our investigations included heel height, insole, and HBS as parameters.

## 2. Materials and Methods

### 2.1. Design Data Sources, Search Strategy, and Study Selection

This systemic review was carried out in accordance with the PRISMA statement [23]. To identify relevant papers, a bibliographical search was conducted in four databases: Web of Science, PubMed, Scopus, and Embase. A manual search was performed in OpenGrey literature in April 2020. In some cases, YDG was responsible for contacting author by e-mail to obtain supplement information. The detailed electronic search was as follows: “high heels”, “high-heeled shoes”, “women's footwear”, “heel height”, “biomechanics”, “comfort height”, “heel base size”, “kinematic parameters”, “kinetic parameters”, “insole measurements”, and “insert”. These keywords are combined and searched on each database. The first and second author (MWZ and CJ) independently performed relevance article screening, which involved the title, abstract, full-text, and data extraction examination.

### 2.2. Eligibility Criteria

The eligibility of selecting papers was estimated according to the following inclusion criteria: (1) the articles had to focus primarily on healthy women wearing HH shoes, (2) the articles were published in English, (3) full-text, peer-reviewed, original scientific articles published in journals, (4) the presented data is associated with HH gait (including spatiotemporal, kinematic, kinetic parameters, and EMG), (5) the articles focused on how to alleviate harmful influences on female health with HH, and (6) the articles had to be retrievable. If the abstract did not present sufficient details for any of the eligibility criteria, the reviewers would browse the full text. Then, if the full text failed to comply with any of the eligibility criteria, it would be deleted.

### 2.3. Data Extraction and Quality Assessment

The important details of the selected articles were extracted by two independent reviewers (ECT and GF). The following data were retrieved from the selected articles: author, year of publication, participant characteristics, shoe condition, measured variables, purpose, and main result. In case of disagreement in data extraction, another reviewer (CJ) was included into the discussion to reach a consensus.

The principles of McMaster Critical Review Form were conducted to thoroughly estimate methodological quality of all selected studies [24–26]. This review form provided 15 separate elements to assess the various types of experimental studies. A 2-point scoring system has been established, where the rating was defined as follows: “yes” (1 point), “no or not measured,” or “not applicable” (0 point). This system can be utilized to appraise whether a study meets the standards for good methodological quality [26].

## 3. Results

### 3.1. Search Results and Validity

The bibliographical database search identified 906 citations: 276 in PubMed, 243 in Scopus, 187 in Web of Science, and 200 in Embase. Duplicates were deleted leaving a total of 362 articles for evaluation. 276 studies were eliminated since after scanning the titles and abstracts of the retrieved papers, it turned out that the content was inconsistent with the standards. 86 full-text studies were extracted for detailed review, and 78 studies were removed as these failed to meet inclusion criteria. A total of 8 studies were eventually eligible for all inclusion criteria. The detailed search strategy is shown in Figure 1, while the basic information of the selected articles is listed in Table 1. Quality evaluation of each article by the McMaster score form is presented in Table 2. All of the extracted papers were graded from moderate to high rating based on the McMaster critical appraisal tool.

### 3.2. Overview of the Included Studies

An accurate recommendation for offsetting negative impact on HH for women is to alter three important parameters, namely, heel height, HBS, and sole insert. The biomechanical investigation of these parameters commonly involve kinematic, kinetic, and perceived stability changes of the lower extremity*, s*uch as plantar pressure in a different region of the foot, COP deviation in a gait cycle, spatiotemporal variation, and comfort rating. One included article contained EMG testing to detect muscle activity in the tibialis anterior (TA), medial gastrocnemius (MG), quadriceps (QUA), hamstrings (HAM), and erector spinae (ES) during walking, and one study recorded heart rate as a physiological variable.

#### 3.2.1. Heel Height

Two studies conducted several experiments to determine an appropriate height heel of high-heeled shoes in order to reduce disturbance of the locomotor pattern. Based on three different walking speeds, Nadège et al. assessed the effect of nine pairs of heel height (0 cm, 2 cm, 3 cm, 4 cm, 5 cm, 6 cm, 7 cm, 8 cm, 9 cm) on kinematic parameters, in which the stride length (SL), swing phase (DSwp), duration of the stance phase (DStp), swing phase (DSwP), and gait ratio were included, as well as heart rate [27]. The results indicated that the most comfortable heel height is 4.13 ± 0.34 cm, which is accompanied with less disruptive locomotor pattern and optimal heart rate, compared to other heights. Differently, Ko and Lee determined the most comfortable heel height for HH shoes by detecting the displacement of the COP and plantar pressure change after walking for 1 hour in 0.5 cm, 4 cm, and 9 cm shoes, respectively [28]. Results presented that 4 cm heel height is the most suitable, since this height is accompanied with stable COP tendency and less plantar pressure than walking in 0.5 cm or 9 cm shoes. Details are presented in Table 3.

#### 3.2.2. HBS

Two studies were associated with the effect of HBS on distribution of plantar pressure patterns, COP trajectory, and perceived comfort. A large HBS demonstrated smaller maximal peak pear pressure in the rearfoot, midfoot, and forefoot compared to small HBS [29, 30]. It must be noted that the scale of HBS affects the COP location in the anterior-posterior direction at the end of the stance phase. The COP deviations are increased with a small HBS when compared to a large HBS [30]. Only one study reported information about the stability as a function of HBS. It can be concluded that a large HBS can lead to a more stable gait during walking with HH [30]. Details are presented in Table 4, and different sizes of HBS are shown in Figure 2(b).

#### 3.2.3. Insert Insole

Four included studies evaluated the effect of insert insole on kinematic, kinetic, EMG, and comfort rating of the lower extremity, but different types of insole were used for each study. One study investigated how subject's rearfoot kinematic, muscle activity, and subjective comfort were affected by TCI which were designed from rearfoot to metatarsal head during walking with HH (Figure 2(b) [31]. When compared with a noninsert condition, results showed that the use of a TCI could reduce peak MG by 19.0% and peak ES by 21.5% in HH with 7.6 cm, and rearfoot inversion angle was significantly decreased. But this study did not present kinetic variation of the foot. Another included article used an insole from the rearfoot to metatarsal head (TCI II) that was designed by the orthotist to fit each participants' foot to determine the effect of shoe inserts on plantar pressure, GRF, and perceived comfort during walking in different heel height shoes (1.0 cm, 5.1 cm, 7.6 cm) (Figure 2(b)) [8]. Results showed that the peak pressure of the medial forefoot reduced by using TCL compared with noninsert shoes, and it was more effective to use TCI in the higher heels than lower and flat heels. Furthermore, Yung and Wei also found that a TCI decreased heel pressure by 25%, medial forefoot pressure by 24%, and impact force by 33% [22].

While the heel cup pad could decrease the heel pressure and impact force and the use of single arch support inserts can attenuate the medial forefoot pressure, no special changes to the metatarsal pad using measured parameters were found [22]. The medial forefoot (MF) has been considered the most sensitive area in response to heel height variation [7, 22, 32, 33]. The effect of four different types of foam insoles (soft 5 mm, soft 10 mm, hard 5 mm, hard 100 mm) in the targeted MF region on plantar pressure was tested. There was a great advantage in soft 5 mm to reduce peak pressure by 26%, impact force by 27% in MF region compared to the noninsert condition [7]. All the above insole types are presented in Figure 2(a). More details on female insert insoles are presents in Table 5.

## 4. Discussion

To reach a full understanding of how the design factors of high-heeled shoes affect locomotor pattern, disturbance of plantar pressure, and perceived comfort is crucial. This review identified 8 articles, which appraised either the effect of heel height, HBS, or insert insole on lower limb kinematic, kinetic, or EMG during waking with HH, as well as perceived comfort.

### 4.1. Heel Height Studies

There are only two studies that evaluated the comfort heel height of HH by using different methods, and a consensus has been formed that shows that the appropriate heel height in high-heeled shoes is 4.13 ± 0.34 cm [27, 28]. In addition, this result is also consistent with Ko who reported that the preferable heel height was between 3 cm and 5 cm, but this article as a conference paper failed to be selected in this review [34]. A growing number of researches indicate that musculoskeletal systems are directly modified from wearing HH. On the other hand, the human foot naturally presents a moderate imbalance in body weight (BW) distribution; i.e., 43% of BW is loaded to the foot front, with the remaining 57% at the heel portion when walking barefoot. For that reason, a slight heel height shoe (2 cm) is recommended to be used by orthopedic specialists, since it can balance the distribution of plantar pressure to relieve rearfoot load [21]. But these outcomes depend on short-term testing rather than for a long period. Therefore, the results of a suitable heel height in included articles may not predict the impact of wearing high-heeled shoes in the long term.

### 4.2. HBS Studies

The scale of HBS is another important factor influencing locomotor pattern during gait with HH. The narrow heels are the most commonly used design in HH which increase plantar pressure, especially in the heel region and lead to instability [22, 35, 36]. Luximon et al. noted that the maximal peak pressure uniformly increased over the whole plantar in large HBS, whereas a narrowed HBS presented higher maximal peak pressure in the toe region [30]. This result is partially similar to Guo et al. whose research showed that the plantar pressure of hallux was significantly increased in small HBS compared to large HBS [29]. Except for the impact of heel height, the narrow HBS may be a direct reason contributing to hammer toe which is caused by excessive pressure on the metatarsal-phalangeal region during walking with HH. Additionally, a smaller HBS presented a larger COP deviation which triggered gait instability, where the toes had to grip the sole of shoes to keep stable. This scenario may be another reason that could lead to the development of a hammer toe when wearing HH [30].

It must be noted that only one heel height was used to measure the function of using different HBS in two selected studies. Although previous researchers suggested that a decreased HBS rather than an increased heel height was the main element for reducing stability during walking with HH [37], the different sizes of HBS combined with diverse heel height should be assessed in the future to further confirm the effectiveness of HBS on gait stabilization.

### 4.3. Insert Insole Studies

Insert insole has been widely used in footwear to improve perceived comfort, absorbing energy attenuating impact forces, redistribute the plantar pressure, and reduce the risk of movement-related injury [38–40]. The various insert designs presented different kinetic modifications during walking with HH. For instance, Yung and Wei indicated that a heel cup pad reduced pressure by 24.3% and impact force by 18.6% in the heel region when wearing HH [22]. An arch support insole decreased peak pressure by 15% in the medial forefoot region and raised the pressure by 125.6% in the midfoot region, since it was used to prevent depression of the longitudinal arch during weight bearing, thereby alleviating the tension of the plantar aponeurosis [22, 41, 42]. Weight bearing can be transferred from the forefoot to the longitudinal and metatarsal arches by the metatarsal pad; however, no changes in pressure and impact forces were found in the medial forefoot region reported by Yung and Wei [22]. Furthermore, medial forefoot pads with different foam hardness and thickness were utilized; and the results showed that the thick soft pad can effectively reduce larger pressure and impact force caused by HH in the medial forefoot when compared to other types [7, 43].

In terms of using TCI, three included studies indicated that TCI relieved pressure and impact force on multiple areas of the foot simultaneously and significantly improved perceived comfort during walking with HH [8, 22, 31]. The TCI provides a highly conforming fit between the foot and the contact surface of the insole, as well as spreading and redistributing pressure over the rearfoot, midfoot, and forefoot. Notably, the current research notes that the use of TCI is the most effective way to attenuate pressure in comparison to other single pads during walking with HH. Further studies are needed to evaluate the effect of different thicknesses and material properties of TCI on load and pressure redistribution during walking with HH shoes. What is more, the effectiveness of insoles also needs to be estimated in the long term to determine whether this type of intervention should be recommended for women with high heel**s-**related foot problems.

### 4.4. Limitations and Future Direction

The most obvious limitation in this review is the small sample size. Only 8 studies met our inclusion criteria hence the reason why a meta-analysis was not conducted. In addition, the effects of walking/running speed on locomotor pattern during high-heeled gait were not studied because there are a wide range of variables and different experimental conditions that would need to be taken into consideration.

It is worth thinking about HH in relation to finite element model analysis and laboratory tests to determine what kind of material properties, hardness, and thickness of insert insole are optimal to minimize the negative impacts of wearing HH. On the other hand, the age, height, and body mass are important parameters in wearing HH; the age affects muscle strength, the height may affect joint moment, and bodyweight directly related to load increase. Future studies should be aimed at providing personal recommendations for HH in terms of choosing the heel height and HBS size based on the individual characteristics that involve weight, height, and age. It seems likely achieved by conducting a comprehensive study that combines the numerical simulation, finite element model analysis, and a large number of sample experiments in the long term.

## 5. Conclusions

We have systematically reviewed studies focused on factors that aim to counter the adverse impacts on high-heeled shoes. The effects of heel height, heel base size, and insert insole on the biomechanical of lower extremity and perceived comfort are concluded. Some evidence demonstrates that (i) the range of appropriate heel height for wearing HH is 3.76 cm to 4.47 cm; (ii) compared to small heel base size, the larger ones effectively increase gait stability, reduce risk of ankle injury, and improve comfort rating during walking with HH; and (iii) the use of a total contact insert significantly decreases plantar pressure and impact forces on the foot so that a higher perceived comfort is achieved. However, there were some limitations in the data presented in the included articles due to the different methodologies used and a limited number of studies. All the above conclusions need to be further tested in a longer duration experiment. In the future, numerical simulation, finite element model analysis, and a large number of sample experiments should be combined to offer personal recommendations for wearing HH based on the individuals' characteristics.

## Figures and Tables

**Figure 1:** Flowchart of the search strategy.

**Figure 2:** (a) The different insert pads mentioned in included studies. (b) The total contact insert, total contact insert II (from rearfoot to metatarsal head), and small and large heel base size mentioned in included studies. Note: (a) and (b) do not represent the actual ones used in the included study.

**Table 1:** Basic information on selected articles.

Number [ref.]	Author/date	Title	Journal	Concentration
1 [27]	Nadège et al. 2015	Wearing high-heeled shoes during gait: kinematics impact and determination of comfort height	American Journal of Life Sciences	Heel height
2 [28]	Ko and Lee 2013	The changes of COP and foot pressure after one-hour walking wearing high-heeled and flat shoes	Journal of Physical Therapy Science	Heel height
3 [30]	Luximon et al. 2015	Effects of heel base size, walking speed, and slope angle on center of pressure trajectory and plantar pressure when wearing high-heeled shoes	Human Movement Science	HBS
4 [29]	Guo et al. 2012	Effect on plantar pressure distribution with wearing different base size of high-heel shoes during walking and slow running	Journal of Mechanics in Medicine and Biology	NBS
5 [31]	Hong et al. 2013	Effect of shoe heel height and total-contact insert on muscle loading and foot stability while walking	Foot and Ankle Society	Insert insole
6 [7]	Li et al. 2010	Biomechanical effects of foam inserts on forefoot load during the high-heeled gait: a pilot study	Journal of Mechanics in Medicine and Biology	Insert insole
7 [8]	Hong et al. 2005	Influence of heel height and shoe insert on comfort perception and biomechanical performance of young female adults during walking	Foot and Ankle International	Insert insole
8 [22]	Yung and Wei 2005	Effects of shoe inserts and heel height on foot pressure, impact force, and perceived comfort during walking	Applied Ergonomics	Insert insole

**Table 2:** Methodological quality of included studies by using the McMaster critical appraisal form.

Number	Study design	Level	Items															Score
			1	2	3	4	5	6	7	8	9	10	11	12	13	14	15	
1	CCT	III-2	√	√	√	√	√	√	x	√	n/a	√	√	√	√	x	√	12/14
2	CCT	III-2	√	√	√	√	√	x	√	√	n/a	√	√	√	√	x	√	12/14
3	CCT	III-2	√	√	√	√	√	x	√	√	n/a	√	√	√	√	√	√	13/14
4	CCT	III-2	√	√	√	√	√	x	√	√	n/a	√	√	√	√	x	√	12/14
5	CCT	III-2	√	√	√	√	√	x	√	√	n/a	√	√	√	√	x	√	12/14
6	CCT	III-2	√	√	√	√	x	x	√	√	n/a	√	√	√	√	√	√	12/14
7	CCT	III-2	√	√	√	√	√	x	√	√	n/a	√	√	√	√	x	√	12/14
8	CCT	III-2	√	√	√	√	√	x	√	√	n/a	√	√	√	√	x	√	12/14

Level of evidence (based on NHMRC hierarchy); CCT: control clinical trial; FU/RCT: follow-up study from randomized control trial. √: yes; x: no/not reported; n/a: not applicable. McMaster Items: (1) study purpose clearly stated; (2) background literature reviewed; (3) appropriate research design; (4) sample described in detail; (5) sample size justified; (6) outcome measure reliability reported; (7) outcome measure validity reported; (8) intervention described; (9) contamination avoided; (10) cointervention avoided; (11) results reported in terms of statistical significance; (12) appropriate analysis method; (13) clinical significance reported; (14) dropouts reported; (15) appropriate conclusion.

**Table 3:** Summary of articles related to the effect of appropriate heel height among females.

Number	Participant characteristics (mean ± standard deviation)				Shoe condition		Walking speed (cm/s)	Variables measured	Purpose	Main findings
	*N*	Age (years)	Height (m)	Weight (kg)	HBS (cm^2^)	Height of heel (cm)				
1	15	22.40 ± 2.56	1.63 ± 0.04	59.07 ± 5.15	5.3	0, 2, 3, 4, 5, 6, 7, 8, 9	0% Ffcwh +20% Ffcwh -20% Ffcwh	(i) SL	To determine the comfort heel height for the shoe	(i) The comfort heel height was 4.13 cm ± 0.34
								(ii) DStP		
								(iii) DSwP		
								(iv) Gait ratio		
								(v) Heart rate		
2	15	20.90 ± 1.30	1.60 ± 3.30	52.10 ± 5.0	—	0.5, 4, 9	1.17	(i) Foot pressure	To determine the most appropriate height for shoe heels	(i) The distribution of foot pressure and COP did not change significantly in 4 cm heel height after walking
								(ii) COP		(ii) 4 cm heel height was preferable for health and comfort

Note: Ffcwh: step frequency freely chosen in shoes without heel; SL: stride length; DStP: duration of the stance phase; DSwP: swing phase; COP: central of pressure.

**Table 4:** Summary of articles related to the effect of HBS on female.

Number	Participant characteristics (mean ± standard deviation)				Shoe condition		Walking speed (cm/s)	Variables measured	Purpose	Main findings
	*N*	Age (years)	Height (m)	Weight (kg)	HBS (cm2)	Height of heel (cm)				
3	15	22.50 ± 4.70	1.61 ± 0.04	51.30 ± 4.90	-0.88, -8.92	3	112, 143	(i) COP	Evaluated the effects of the HBS of HH shoes	(i) Smaller COP deviations in larger HBS
								(ii) Perceived stability		(ii) The walking speed mainly affected the locations of the COP in the anteroposterior direction during gait
								(iii) Plantar pressure		(iii) A maximal peak pressure increased over the forefoot, midfoot, and rearfoot in larger HBS
										(iv) The participants felt more stable in larger HBS
4	13	22.0 ± 0.8	1.60 ± 3.30	52.10 ± 5.0	-1.44, -7.7	7.8	100, 115, 200	(i) Plantar pressure	Be better to select one with a wide-based heel	(i) Smaller plantar pressure in medial, central, and lateral of forefoot and toe regions in larger HBS

Note: COP: central of pressure; HBS: heel base support; HH: high heels.

**Table 5:** Summary of articles related to the effect of insert insole on female.

Number	Participant characteristics (mean ± standard deviation)				Shoe condition	Type of insole	Variables measured	Purpose	Main findings
	*N*	Age (years)	Height (m)	Weight (kg)	Height of heel (cm)				
5	15	24.5 ± 4.5	159.3 ± 6.5	49.6 ± 6.4	1.0, 5.1, 7.6	(i) TCI II (from rearfoot to metatarsal head)	(i) Kinematic (ii) EMG (iii) Comfort rating	To investigate how shoe heel height and use of TCI in high-heeled shoes affect the wearer's rearfoot complex, muscle loading, and subjective comfort	(i) The use of TCI reduced the rearfoot inversion angle and in both QUA and ES muscles activity (ii) Comfort rating increased by using TCI
6	8	22.0 ± 2.0	163.0 ± 3.0	51.0 ± 4.5	0, 4.5, 8.5	(i) MF foams insole with soft (5 mm), (ii) MF soft 10 mm (iii) MF hard 5 mm (iv) MF soft 10 mm	(i) Plantar pressure	To determine the effect of foam inserts in targeted medial foot region on the foot pressure distribution during normal walking	(i) Thicker soft foam sole significantly reduced peak pressure in MF than thinner hard foams (ii) The maximum force and peak pressure reduced in the MF region bu using foams than no insole in HH
7	20	25.4 ± 3.8	157.8 ± 5.0	50.5 ± 4.2	1.0, 5.1, 7.6	(i) TCI insole	(i) Perceived stability (ii) Plantar pressure (iii) GRF	To evaluate the effect of TCI on comfort perception and plantar pressure	(i) The comfort ratings were significantly increased when wearing with TCI (ii) Use of the TCI reduced the peak pressure in the medial forefoot (iii) Mean GRF decreased to 39% BW in the highest shoes with the TCI (iv) It was more effective to use TCL in higher heels than in the lower heels and in flat heels
8	10	23 ± 3.4	160 ± 3	50 ± 3	1.0, 5.1, 7.6	(i) Heel cup pad (ii) Arch support (iii) Metatarsal pad (iv) TCI	(i) Plantar pressure (ii) Comfort rating	Whether use of shoe inserts change foot pressure distribution, impact force, and perceived comfort during walking	(i) Heel cup insert reduced the heel pressure and impact force (ii) Arch support insert reduced the medial forefoot pressure and improved comfort (iii) TCI reduce heel pressure, medial forefoot pressure, and impact force and provided a higher perceived comfort

Note: TCI: total contact insert; MF: medial forefoot; GRF: grand reaction force; BW: body weight; QUA: quadriceps; ES: erector spinae; EMG: electromyography.
